# Employment of Alginate Floating *In Situ* Gel for Controlled Delivery of Celecoxib: Solubilization and Formulation Studies

**DOI:** 10.1155/2020/1879125

**Published:** 2020-05-31

**Authors:** Bazigha K. Abdul Rasool, AlZahraa Khalifa, Eman Abu-Gharbieh, Rawoof Khan

**Affiliations:** ^1^Pharmaceutics Department, Dubai Pharmacy College for Girls, Dubai, UAE; ^2^Clinical Sciences Department, College of Medicine, University of Sharjah, Sharjah, UAE; ^3^Dubai Institute for Environmental Research and Laboratory Analysis, Dubai, UAE

## Abstract

Celecoxib (CXB) is a COX-2-selective nonsteroidal anti-inflammatory drug used to control pain and various inflammatory conditions. CXB has limited oral bioavailability and a slow dissociation rate due to its poor water solubility. In order to enhance the oral bioavailability of CXB and reduce the frequency of administration, the present study was aimed at enhancing the aqueous solubility of CXB by a cosolvency technique and then at formulating and evaluating a CXB *in situ* floating gelling system for sustained oral delivery. Three cosolvents, namely, PEG 600, propylene glycol, and glycerin, at different concentrations, were used to solubilize CXB. Particle size analysis was performed to confirm the solubility of CXB in the solutions. The floating *in situ* gel formulations were then prepared by the incorporation of the CXB solution into sodium alginate solutions (0.25, 0.5, and 1% *w*/*v*). Formulations, in sol form, were then *in vitro* characterized for their physical appearance, pH, and rheological behaviors, while formulations in gel form were evaluated for their floating behavior and *in vitro* drug release studies. FTIR spectroscopy was performed to examine drug-polymer interaction. The selected formula was evaluated biologically for its anti-inflammatory and analgesic activities. Results revealed that the less-polar solvent PEG 600 at 80% *v*/*v* had the highest solubilization potential, and it was used to optimize the *in situ* gel formulation. The candidate formula (F3) was found to have the highest sodium alginate concentration (1% *w*/*v*) and showed the optimum sustained release profile with the Higuchi model release kinetics. The results from the FTIR spectroscopy analysis showed noticeable drug-polymer molecular interaction. Moreover, F3 exhibited a significantly higher percentage of paw edema inhibition at 8 h compared with the reference drug (*p* < 0.05). Also, it showed a sustained duration of analgesia that persisted for the entire experimental time.

## 1. Introduction

Celecoxib (CXB), a selective COX-2 inhibitor, is a nonsteroidal anti-inflammatory drug used primarily for the treatment of various inflammatory and painful conditions [1]. Currently, the available dosage forms of CXB are intended only for oral administration. However, the oral absorption of CXB is limited with a bioavailability ranging from 22 to 40% [2]. According to the Biopharmaceutics Classification System (BCS), CXB is classified as a Class II drug that is practically insoluble at pH conditions in the gastrointestinal tract [3]. The extremely low water solubility of CXB is related to many formulation problems and limits its therapeutic efficiency by delaying the rate of absorption and onset of action. Therefore, it is essential to improve its solubility as it is a potential candidate for advanced solubilization techniques.

The literature reported various solubilizing techniques to improve the solubility and oral absorption of CXB, such as a self-emulsifying system [4], mesoporous silica [5], nanosuspension [6, 7], elixir [8], and solid dispersion [9]. Nevertheless, in previous studies, no attempt has been taken to investigate the aqueous solubility enhancement of CXB by the cosolvency approach.

On the other hand, due to several variables that change throughout the gastrointestinal tract which significantly affect drug absorption, it is evident that the conventional drug delivery system does not easily overcome the difficulties imposed by the gastrointestinal system.

For instance, the incomplete dissolution of the drug and the associated reduction of dose effectiveness are consequences of the incapacity of the conventional drug delivery system to be retained at the stomach level [10]. Therefore, there is a need to develop a sustained release dosage form that can improve the oral bioavailability of CXB and also reduce repeated administrations.

In order to overcome these challenges, technological researchers have developed pharmaceutical systems that control drug release and the residence time, some of which are already available on the market. Gastroretentive drug delivery systems are a good example; they emerged to enhance the bioavailability and effectiveness of drugs with a narrow absorption window.

The *in situ* gelling systems have become more distinguished among the various novel drug delivery systems. These are polymeric formulations that are in sol forms before entering the body but change to gel forms under the physiological conditions such as pH change, temperature modulation, or solvent exchange [11].

Numerous advantages of the *in situ* gelling system, such as stability, biocompatibility, reproducibility, ease of application, and reduced frequency of administration, make the *in situ* gel dosage form more attractive for commercial use [11]. Moreover, the *in situ* gel dosage form would improve patient compliance and comfort, exhibit sustained and controlled rates of absorption and excretion, and possess a reasonable margin of safety [12].

Various natural and synthetic polymers are currently used for oral, buccal, rectal, vaginal, ocular, intraperitoneal, and parenteral *in situ* gel formulation. Pectin, xyloglucan, gellan gum, chitosan, and alginic acid are some of the natural polymers [13].

This study is aimed at developing a CXB *in situ* gel system for sustained oral drug delivery using natural biodegradable polymers and the cosolvency technique to enhance the aqueous solubility of CXB and at evaluating the bioactivity of the prepared formula on animal models.

## 2. Materials and Methods

### 2.1. Materials

CXB BP was purchased from Sigma-Aldrich, USA. Polyethylene glycol (PEG 600), propylene glycol (PG), and glycerin were from Alpha Chemika, India. Sodium alginate (SA) (Fluka) 90 cps (1% *w*/*v* solution in water at 25°C) and calcium chloride (CaCl_2_) (E. Merck, India) were used. All other reagents were of analytical grade.

### 2.2. Estimation of CXB

CXB estimation was performed spectrophotometrically at *λ*_max_ of 252 nm using a UV-1800 UV-VIS spectrophotometer (Shimadzu, Japan). The stock solution was prepared in methanol at a 1000 *μ*g/mL strength, and the drug's absorbance was recorded against the blank, methanol. The calibration curve was prepared at concentration ranges between 6 and 24 *μ*g/mL to estimate the drug content [14]. The method was validated for linearity, accuracy, and precision. The experiments were repeated three times to check its reproducibility. CXB absorbance was measured as a mean ± SD (*n* = 3). The regression equation for the calibration curve was generated from the linear regression analysis on a Microsoft Excel worksheet 2010 and was later used for the determination of CXB concentration.

### 2.3. Solubility Studies

Excess amount of CXB pure powder was added to mixtures of distilled water and cosolvents (PEG 600, PG, and glycerin) at various concentrations (0, 20, 40, 60, 80, and 100% *v*/*v*). The mixtures were placed in conical flasks and closed well with stoppers. The flasks were shaken using a Thermo Scientific Precision SWB-15 shaking water bath at a shaking speed of 50 rpm and temperature of 25 ± 0.5°C for 48 h to obtain equilibrium [15]. Then, aliquots were withdrawn, filtered through a Millipore® filter membrane (0.45 *μ*m pore size), and diluted appropriately. The samples were analyzed using a UV-1800 UV-VIS spectrophotometer (Shimadzu, Japan) at 252 nm wavelength, and the solubility of CXB (mg/mL) in each sample was determined.

### 2.4. Particle Size of CXB-Cosolvent Mixture

The particle size was measured in a range of 0.1 nm and 10 *μ*m by using a Malvern® Zetasizer. Particle size measurement was used at the point of maximum solubility. One millilitre of each sample was diluted up to 10 mL with distilled water (1 : 10 *v*/*v*) and filtered through a Millipore® membrane filter (pore size 0.45 *μ*m). Samples were then placed in a capillary measurement cell, and particle size analysis was carried out at 25°C.

### 2.5. Preparation of CXB *In Situ* Floating Gel Formulations

Three formulas of the CXB *in situ* floating gel were prepared by dispersing the CXB powder thoroughly in SA solutions (0.25%, 0.5%, and 1%*w*/*v*). SA aqueous solutions were prepared by heating to 60°C with continuous stirring followed by cooling to 40°C. Then, CaCl_2_ (cross-linking agent), CaCO_3_ (gas-forming agent), citric acid, and sodium citrate were added to the mixture. The composition of CXB floating *in situ* gel formulations is shown in Table 1.

### 2.6. *In Vitro* Characterization of CXB *In Situ* Gels

#### 2.6.1. Physical Appearance and pH

The color and the clarity of the floating *in situ* gel formulations were evaluated by the visual inspection of the sols against a dark and white illuminating background. The pH of the formulas was measured in triplicate using an Edge HI2002-01 pH meter (Hanna Instruments) at room temperature.

#### 2.6.2. Rheological Behavior

The prepared formulas were placed inside a sample adaptor of a Brookfield DV-III Ultra Rheometer. The rheological behavior of the gel formulations was examined at different angular velocities (10, 20, 30, 50, 60, and 100 rpm) by using a spindle no. S27. The viscosity was determined at 25°C, as a mean ± SD of triplicate measurements.

#### 2.6.3. Floating Behavior

The floating behavior was determined by observing the floating lag time (FLT), the time taken for the formula to emerge to the surface of the medium, and the duration of floating (DOF), the time the formula constantly floated on the medium surface for each formula. The *in vitro* gelling capacity was graded in three categories based on FLT and DOF [15], as follows:

*Low gelling capacity (+)*: FLT (immediate gelation) and DOF < 12 h

*Intermediate gelling capacity (++)*: FLT (immediate gelation) and 24 h > DOF > 12 h

*High gelling capacity (+++)*: FLT (immediate gelation) and DOF > 24 h

This study was performed by placing an accurately weighed sample (1 g) of each formula in a test tube containing 10 mL of the simulated gastric fluid USP without pepsin enzyme (constituents: 2 g NaCl and 7 mL HCl in D.W. to make 1 L), and samples were then observed for their floating behavior.

### 2.7. *In Vitro* Drug Release

The *in vitro* release of CXB from the formulations was determined using a USP dissolution apparatus type II (paddle). The vessels were filled with 900 mL of the dissolution medium (0.1 N HCl, pH 1.2). The temperature was maintained at 37 ± 0.5°C, and the operating speed was 50 rpm [16]. Samples of 5 mL were withdrawn at 0.5, 1, 2, 3, 4, 5, 6, 7, and 8 h and replaced with the same volume of the fresh buffer to maintain the sink condition. The drug content in samples was determined as a cumulative percentage release by using a UV-1800 UV-VIS spectrophotometer (Shimadzu, Japan) at 252 nm.

To understand the mechanism of CXB release from the *in situ* gels, the *in vitro* dissolution data of the prepared formulas were fitted to different kinetics models, including first-order kinetics, zero-order kinetics, the Higuchi model, and the Korsmeyer-Peppas model [17]. The release rate constants and correlation coefficients (*R* ^2^) were obtained from the linear regression analysis on Microsoft® Excel 2013.

### 2.8. FTIR Spectroscopy Analysis

Samples (10 mg) of CXB powder, SA powder, CXB/SA physical mixture, and freeze-dried gel were loaded into a Shimadzu FTIR spectroscope (IRAffinity-15, Japan), and their spectra were recorded over a wave range of 450-4000 cm^−1^. The CXB-loaded SA gel was dried by a Biobase Freeze Dryer (BK-FD10P, China) under the conditions of -59°C and 0.001 mp vacuum pressure for 24 h.

The CXB/SA physical mixture was prepared by continuous mixing in a mortar and pestle of CXB with the polymer at a molar ratio of 1 : 1 *w*/*w* for 30 min. FTIR spectroscopy analysis was performed to study the possibility of the molecular interaction between CXB and SA.

### 2.9. Biological Evaluation

#### 2.9.1. Experimental Animals

Thirty-six adult, healthy Wistar albino rats of both sexes weighing 150 g-200 g, approximately two months old, were used for the biological evaluation studies. The animals were maintained under standard conditions, fed with regular diet and water supplied *ad libitum*, and accommodated for seven days before the experiments. The experimental protocol followed the ethical standards for laboratory animals [18] and was approved by the Ethical Research Committee of Dubai Pharmacy College, Dubai, United Arab Emirates.

#### 2.9.2. Experimental Protocol

Based on the *in vitro* results, the best formula was selected to proceed to the *in vivo* evaluation. Animals were randomly divided into six groups of six animals each. The first three groups were used for the anti-inflammatory activity evaluation, and the others were used for the analgesic test.

In each experiment, the first group of animals served as the control and received oral saline. The second group served as a positive control group and received a 50 mg/kg dose of the reference drug, Celebrex® capsules, orally, and the third group received the F3 formula orally at a dose of 25 and 50 mg/kg.

#### 2.9.3. Anti-Inflammatory Activity

Carrageenan-induced paw edema in the rats' test was used to assess the acute anti-inflammatory activity of the developed formula. One-hour posttreatment, the inflammation was induced by injection of 0.1 mL of 1% (*w*/*v*) carrageenan solution into the left hind paw of each rat. The baseline paw volumes of all animals were recorded using a LE7500-digital plethysmometer (Harvard, USA). The relative increase in paw volume was determined by measuring the paw volume after 1, 3, 5, and 8 h, following the carrageenan administration [19]. The percentage inhibition of edema was compared with the controls. The percentages of inhibition were obtained using the following formula:

(1) $$\begin{array}{c} \text{Percentage of inhibition}=\frac{\left(V_{t}-V_{0}\right)\text{control}-\left(V_{t}-V_{0}\right)\text{treated}}{\left(V_{t}-V_{0}\right)\text{control}}\times 100, \end{array}$$

where *V*_*t*_ and *V*_0_ are the average volumes for each group posttreatment and pretreatment, respectively.

#### 2.9.4. Analgesic Effect

Thirty minutes before treatment, 1% *w*/*v* carrageenan suspension (0.01 mL) was injected into the supplanter area of the right hind paw of the animal. In the test, the rat was placed on a hot plate maintained at 55 ± 0.5°C. The time elapsed until the occurrence of either a hind paw licking or a jump off the surface was recorded as the hot plate latency. The animals were tested at 0, 0.5, 1.0, and 3.0 h. The cut-off time was 50 s to prevent tissue damage, and mice with baseline latencies of <5 were eliminated from the study [20].

### 2.10. Statistical Analysis

The measurements were expressed as mean values along with their standard deviations. For the *in vitro* studies, the statistical assessment was conducted using the analysis of variance followed by Bonferroni's correction for multiple comparisons. A *p* value < 0.05 was considered significant. Calculations were performed using GraphPad Prism Software Version 6.

## 3. Results and Discussion

### 3.1. CXB Calibration Curve

CXB calibration curve was prepared by plotting the mean absorbance ± SD of CXB in the diluted solutions against their relevant concentrations (Figure 1). Linear regression of absorbance on concentrations gave the equation *y* = 0.0426*x* with a correlation coefficient (*R* ^2^) of 0.999. The high value of *R* ^2^ indicated that the concentrations used in the preparation of the calibration curve were convenient and in compliance with Beer's law.

### 3.2. Solubility of CXB

Basically, the addition of a cosolvent is an effective technique to enhance the solubility of poorly soluble drugs [21, 22]. Cosolvents are water-miscible solvents, commonly used in pharmaceutical manufacturing to enhance drug solubilization. The nonpolar hydrocarbon region within the cosolvent reduces the ability of the aqueous system to repel nonpolar solutes. In the present study, three widely used cosolvents, PEG 600, PG, and glycerol, were evaluated for the aqueous solubility of CXB. The cosolvent with higher drug solubility in the pure state is referred to be the stronger solvent.

CXB has a very poor solubility in water that is attributed to a predominantly nonpolar feature of its molecule structure (Figure 2). The solubility of CXB in various water-cosolvent mixtures with their respective dielectric constants is represented in Table 2. Results indicated an inverse relationship between CXB solubility and solvent polarity. The cosolvent efficiency ratio, i.e., the ratio of solubility of a drug in a cosolvent-water mixture to the solubility of the drug in water without PEG 600, PG, and glycerol (80% *v*/*v*), was found to be 1383.6, 884.5, and 184.5, respectively. This is probably because of extensive hydrophobic interactions between the drug and the solvent.

The dielectric constants of the solvent mixtures were calculated by the following formula:

(2) $$\begin{array}{c} \varepsilon_{\text{mix}}=\varepsilon_{\text{ws}}f_{\text{ws}}+\varepsilon_{\text{ss}}f_{\text{ss}} \end{array}$$

where *ε* and *f* are the dielectric constant and volume fraction, respectively, and the subscripts mix, ws, and ss represent values for the mixture, weaker solvent, and stronger solvent, respectively.

Solubility usually increases with a decrease in the dielectric constant of the mixture. However, a considerable reduction in CXB solubility was achieved by using the cosolvents alone compared with 80% *v*/*v* of cosolvent-water mixtures. This effect occurs because CXB has some degree of polar property as well and maximum solubilization related to the polarity of the solute and the solvent.

In addition, the solubility in a water-cosolvent mixture (Sm) was calculated from the solubility values in pure water (Sw) and in the neat cosolvent (Sc) and the volume fraction concentrations of water and the cosolvent, fw and fc, respectively, in the solvent mixture

(3) $$\begin{array}{c} \log\text{ Sm}=\text{fc}\log\text{ Sc}+\text{fw}\log\text{ Sw}. \end{array}$$

Therefore, the solubilization of hydrophobic drugs in water-cosolvent mixtures was represented by the log-linear model [23] that is expressed sometimes using the solubilization power of the cosolvent (*σ*) as follows:

(4) $$\begin{array}{c} \log\text{ Sm}=\log\text{ Sw}+\sigma \text{fc}, \end{array}$$

where *σ* = log(Sc/Sw) is the solubilization power of the cosolvent.

The solubility data of CXB in the water-cosolvent mixtures were used to plot a log-linear solubilization curve, as shown in Figure 3. Results revealed that the maximum cosolvent solubilizing effect of the three cosolvents was obtained at the concentration of 80% *v*/*v*. PEG 600 80% *v*/*v* showed the highest solubilization potential produced the highest solubility of CXB (3.044 ± 0.0552 mg/mL) compared to the other two cosolvents, PG and glycerol. Solubilization powers (*σ*) of PEG 600, PG, and glycerol cosolvents were calculated by regression analysis from the log-linear solubilization plot and found to be 3.0563 (*R* ^2^ = 0.9999), 2.8939 (*R* ^2^ = 0.9955), and 1.4435 (*R* ^2^ = 0.9853), respectively, since the cosolvents act by decreasing the density of the hydrogen bonds of water, thus creating a less-polar environment in the mixture that enhances the miscibility of drug molecules in the solution. As predicted, PEG 600 being less-polar exhibited the highest (*p* < 0.05) solubilization power compared to propylene glycol and glycerol. The chemical structure of PEG 600, H-[O-CH_2_-CH2]n-OH, facilitates its miscibility in water through the formation of hydrogen bonds. Moreover, PEG 600 has a high surface tension (44.6 dyne/cm at 20°C) and wide dielectric constant ranges. With the help of the hydrophobic hydrocarbon region of CXB, hydrogen bonds between water were broken, thus allowing the hydrophobic compounds to fit in [24].

### 3.3. Particle Size Analysis

The particle size was determined in a range between 0.1 nm and 10 *μ*m using a Malvern® Zetasizer. The mean particle size and polydispersity index (PDI) values for three samples prepared with PEG 600 at different concentrations 40, 60, and 80% *v*/*v* were 538.1 nm ± 62.12 (0.57), 256.1 nm ± 6.652 (1.00), and 235.3 nm ± 16.42 (0.16), respectively. The smallest particle size of CXB, a narrow size distribution, was achieved with 80% PEG solution indicating the maximum solubility of CXB (Figure 4). Knowing that the PDI value describes the degree of nonuniformity of the size distribution of particles within a sample, this index is dimensionless and scaled such that the PDI value preferred to fall in the range of 0.05-0.7, which practically indicates a suitable degree of homogeneity of the sample [25].

### 3.4. Physical Appearance and pH of the *In Situ* Gel

Based on the obtained results, CXB solubilized in 80% *v*/*v* of PEG 600 in water was selected to prepare the *in situ* gel. All the prepared SA-based *in situ* gels of CXB were clear and homogenous. The mean pH values of the formulations in the form of the sol system were in the range of 5.63-6.13 (Table 3). A citrate buffer was added to the formulations to maintain their pH values relatively constant in the gastric medium. Consequently, it might ensure safety and compatibility of the formulations with the biological system in the form of an oral dosage form [26].

### 3.5. Rheological Behavior

Results revealed that viscosity of the prepared sols was directly related to the concentration of SA. The highest value of viscosity was shown by F3 (562.5 ± 17.68 cp) followed by F2 (237.5 ± 17.68 cp) and F1 (137.5 ± 17.68 cp), at a shear rate of 3.4 S^−1^ (10 rpm). However, increasing the shear rate to 34 S^−1^ (100 rpm) resulted in a significant (*p* < 0.05) decrease in the viscosity of all formulas (F3: 207.5 ± 6.35 cp, F2: 74 ± 1.41 cp, and F1: 38.75 ± 1.77 cp) (Figure 5(a)). Viscoelastic fluids exhibit high viscosity under a low shear rate and vice versa. This kind of rheological behavior is more preferred in pharmaceutical preparations since it helps the easy administration of sol preparations at the site of administration followed by conversion into a gel structure *in vivo* which is desirable for release sustainability of the drug [27]. Further data analysis was performed via the preparation of rheograms by plotting the shear rate (S^−1^) vs. shear stress (Pas) to grasp the formulas' flow behavior. All formulas showed a non-Newtonian plastic rheological behavior where a certain amount of force must be applied to the fluid before the induction of any flow. This force is called the yield value. Once the yield value is exceeded and flow begins, plastic fluids may display a Newtonian flow. F3 presented the highest yield value comparing to F1 and F2 (Figure 5(b)). Moreover, all the prepared sols showed convenient flow properties and acceptable pourability, which is necessary to ensure ease of drug administration to the patient.

### 3.6. Floating Behavior

All the prepared formulas showed instant gelation upon contact with the simulated gastric fluid. The floating lag time varied with the formulation variables. F1 exhibited the least FLT (8.32 s), while F3 had the highest lag time (22.5 s). The fast buoyancy behavior of the formulas can be attributed to the presence of the floating agent, calcium carbonate, in the formulations as an insoluble dispersion. Hydrochloric acid, the key component of the gastric juice, reacted with calcium carbonate and formed CaCl_2_, water, and CO_2_ gas. CaCl_2_ is highly soluble in the aqueous solution (74.5 g/100 mL at 20°C) and is ionized in the solution to form Ca^+2^ and Cl^−2^ ions [28]. Ca^+2^ ions also ensued from the ionization of CaCl_2_, a cross-linking agent in the formulations. These ions were capable to cross-link SA molecules and form the double-helical three-dimensional network structure of the gellious matrix, while the released CO_2_ gas got entrapped in the gel and resulted in floating of the matrix.

DOF of F3 was more than 12 hs but less than 24 hs, while F1 and F2 maintained the gel structure for longer than 24 h (Figure 6). The buoyancy behavior of F3, the longest FLT and shortest DOF, can be imputed to the increase in the SA content in the formulation, which consequently made the floating more difficult for the shortened time. However, all formulas presented good gelation capacity (Table 3), which is advantageous, since the drug sol is promptly converted into a thick gel matrix which floated over the stomach juice and worked as a reservoir releasing the drug in a sustained manner during the course of therapy [29]. In some previous studies, the gelation code (+++) indicated that “gelation” was immediate and retained its integrity for an extended period of time; however, the gel was stiff which may cause irritation and discomfort to the patient while (++) demonstrated the optimum gelation characteristics [30, 31].

### 3.7. *In Vitro* Drug Release

The amount of CXB released in the dissolution medium was determined from the regression line equation, *y* = 84.132*x* − 0.0068 (*R* ^2^ = 0.9994), which was obtained from the previously prepared calibration curve of CXB in 0.1 N HCl at *λ*_max_ 233. The concentration of SA was found to be essentially affecting the pattern of the drug's release. The cumulative amount released by CXB significantly (*p* < 0.05) decreased with the increment of the polymer's concentration. This could be due to either the entrapment of CXB inside the networks of the gel's matrix or the polymer-drug molecular interaction. Similar results were also reported in previously published research works [32]. Despite F1 releasing the highest amount of CXB during the first half an hour of the test compared to F2 and F3, the optimum sustained drug release profile till the end of the run was practiced by F3, as shown in Figure 7. Moreover, the amount of CXB released from all formulas was significantly (*p* < 0.05) much higher than that of the reference drug (Celebrex® capsule by Pfizer, dose: 200 mg of CXB). This improvement in drug release can be attributed to the efficiency of the used technique, cosolvency, for CXB solubilization.

The kinetics modeling study on *in vitro* drug release revealed that the Higuchi model was superior in describing the *in vitro* release of CXB from the optimized formulation, F3, as shown in Table 4. In addition, the mechanism of the drug's release for all formulas was found to be a Fickian diffusion release since the *n* value of all formulas was ≤0.5 [33]. Thus, the flux of CXB from the delivery system to the dissolution medium is basically controlled by the gel's matrix's thickness and the concentration gradient across a specified sectional area.

### 3.8. FTIR Spectroscopy

Figure 8 represents the FTIR spectra of CXB, SA, CXB/SA physical mixture, and CXB dried gel. In IR spectra, CXB showed medium absorption bands at 3229 cm^−1^ and 3334 cm^−1^, which were assigned to the drug-NH symmetric and asymmetric stretching vibrations of the primary amine group. The other characteristic bands may be attributed to the following group vibrations: a strong peak at 1738 cm^−1^ (N-H bending), 1445 and 1497 cm^−1^ (S=O symmetric and asymmetric stretching, respectively), and 791 cm^–1^ (aromatic –CH bend). The FTIR spectra of SA pure powder showed stretching vibrations of the O-H functional group at wavenumbers 3200-3400 cm^−1^, and peaks at 1404 cm^−1^ and 1597 cm^−1^ were attributed to asymmetric and symmetric stretching vibrations of carboxylate salt ion, respectively, in addition to the mannuronic acid functional group at wavenumber 884 cm^−1^ and the uronic acid at wavenumber 1025 cm^−1^.

In the IR spectrum of the CXB/SA physical mixture, CXB peaks were prominent than SA, which seems superimposed by CXB. Moreover, the spectrum showed the absence of major peaks, the N-H bending vibration (1738 cm^−1^) of the amine functional group and the O-H stretching vibrations (3200-3400 cm^−1^) of the carboxylic group, which were present in the spectrum of CXB and SA powders alone, respectively. On the other hand, changes in the spectrum of the gel sample were more noticeable than in the physical mixture (Figure 8). There was a decrease in the intensity of carboxylate peaks at 1404 cm^−1^ and 1597 cm^−1^ in the gel spectrum compared to the pure component, which could be due to alginate cross-linking by calcium ions to form the egg-box structure of the gel [34]. The spectrum exhibited changes in the peaks of both CXB and SA, confirming the molecular interaction of CXB with SA in the gel. These findings strongly supported the idea of intermolecular hydrogen-bonding between the C=O group of SA and the (–NH_2_) group of the sulfonamide substituent in the CXB molecule. Hydrogen bonding between SA and chemical compounds was also reported in previous studies [35, 36]. On the contrary, the ionic drug-polymer interaction had unlikely formed, as CXB is a weak organic acid (pKa = 11.1) that predominantly exists in the unionized form at pH values below its pKa.

### 3.9. *In Vivo* Evaluation in Animals

#### 3.9.1. Anti-Inflammatory Activity

The optimized floating *in situ* gel formula of CXB (F3) has shown significant inhibition of carrageenan-induced rat paw edema from 2 to 8 hrs in rats following oral administration, as compared with the control and standard group of animals (Figure 9). The highest percentage of inhibition of the standard drug was found to be 75.83% (*p* < 0.05), whereas the optimized floating *in situ* CXB gel formula (F3) has 92.64% inhibition of paw edema at 8 h (*p* < 0.05), as shown in Table 5. Although the standard drug showed significant inhibition of paw edema, the optimized floating *in situ* gel showed a higher percentage of inhibition at 8 h.

#### 3.9.2. Analgesic Activity

The results of the analgesic activity test are represented in Table 6. Formulation F3 showed high and persistent analgesic activity starting from 0.5 h till the end of the 3 hours (*p* < 0.001) compared to the reference drug that showed the maximum activity after one hour (*p* < 0.05). F3 formulation, with a sustained release pattern, ensured the prolonged duration of analgesia that persists for the entire experimental time.

## 4. Conclusion

The present study evaluated and compared the aqueous solubility enhancement of CXB using three different cosolvents, namely, polyethylene glycol (PEG 600), propylene glycol (PG), and glycerin. PEG 600 80% *v*/*v* was selected in terms of the most efficient solubilizing cosolvent and particle size distribution. The CXB formulated as a floating *in situ* gel containing 1% SA is a potential candidate for the oral administration of CXB that can provide a sustained release pattern with Higuchi model kinetics. FTIR spectroscopy analysis proved a considerable interaction between CXB and SA molecules, which played a significant role in modifying the drug release from the gel delivery system. The candidate formulation F3 showed high and persistent analgesic and anti-inflammatory activities in rats compared to the commercial reference product.

## Figures and Tables

**Figure 1:** Calibration curve of CXB in methanol (mean ± SD, *n* = 3).

**Figure 2:** Chemical structure for CXB.

**Figure 3:** Log-linear solubilization plot of CXB in different cosolvent mixtures (mean ± SD, *n* = 3).

**Figure 4:** Particle size distribution curve by the intensity of CXB in PEG 600 80% *v*/*v*.

**Figure 5:** (a) 3D-surface plot of viscosity and shear stress as a function of shear rate for F1, F2, and F3. The graph was prepared by Minitab® 19. (b) Rheograms of the sol systems (F1, F2, and F3); the viscosity is given as a mean ± SD (n = 3) at 25°C.

**Figure 6:** Floating behaviors of F1, F2, and F3 *in situ* gels in the simulated gastric medium after 1 h and 24 hs.

**Figure 7:** *In vitro* drug release from alginate-in situ gel formulations compared with the reference product (mean ± SD, *n* = 3).

**Figure 8:** FTIR spectra of CXB powder, SA powder, physical mixture, and CXB-dried gel. Color legend indicates the following: black: CXB; blue: SA; pink: CXB/SA physical mixture; and green: CXB-dried gel.

**Figure 9:** Effect of CXB on carrageenan-induced rat paw edema at different time intervals. Results are given as mean ± SEM (*n* = 6), ^∗^Significant effect at *p* < 0.05.

**Table 1:** Composition of CXB floating *in situ* gel formulations.

Ingredients (% *w*/*v*)	F1	F2	F3
CXB	0.6	0.6	0.6
SA	0.25	0.5	1.0
Calcium chloride	0.15	0.15	0.15
Calcium carbonate	0.5	0.5	0.5
Citric acid	0.1	0.1	0.1
Sodium citrate	1.0	1.0	1.0

**Table 2:** Solubility profile of CXB in water-PEG 600, PG, and glycerol mixtures at 25°C.

Water (% *v*/*v*)	Cosolvent (% *v*/*v*)	PEG 600		PG		Glycerol	
		DC	CXB (mg/mL)	DC	CXB (mg/mL)	DC	CXB (mg/mL)
0	100	11.60	2.898 ± 0.0828	32.00	1.860 ± 0.0448	42.50	0.395 ± 0.0196
20	80	24.95	3.044 ± 0.0552	41.27	1.946 ± 0.0383	49.67	0.406 ± 0.0153
40	60	38.30	0.741 ± 0.0312	41.27	0.637 ± 0.0175	56.84	0.265 ± 0.0072
60	40	51.66	0.177 ± 0.0098	50.54	0.164 ± 0.0072	64.02	0.112 ± 0.0048
80	20	65.00	0.045 ± 0.0043	95.82	0.036 ± 0.0032	71.19	0.059 ± 0.0032
100	0	78.38	0.0022 ± 0.002	78.36	0.002 ± 0.0018	78.36	0.002 ± 0.0032

DC: dielectric constant (*ε*); results are given as mean ± S.D. (*n* = 3).

**Table 3:** pH value and floating behavior of CXB *in situ* gels^∗^.

Formulation code	F1	F2	F3
pH	5.65 ± 0.106	6.14 ± 0.035	6.21 ± 0.064
FLT (sec)	8.32 ± 0.009	9.34 ± 0.047	22.5 ± 0.201
DOF (h)	>24	>24	24 h > DOF > 12 h
Gelation capacity	+++	+++	++

^∗^Results are presented as mean ± SD (*n* = 3).

**Table 4:** Results of curve fitting of the *in vitro* diclofenac sodium release data from different optimized alginate-PVP K30 microbeads.

Formula code	Zero-order kinetics		First-order kinetics		Higuchi model	Korsmeyer-Peppas model			
	*K*_o_ (% h^−1^)	*R* ^2^	*K*_1_ (h^−1^)	*R* ^2^	*K*_*H*_ (% h^-1/2^)	*R* ^2^	*K*_KP_ (% h^−1^)	*n*	*R* ^2^
F1	4.456	0.625	0.097	0.4286	24.116	0.6332	45.245	0.216	0.505
F2	2.547	0.167	0.086	0.019	24.087	0.6536	41.264	0.325	0.601
F3	2.308	0.209	0.027	0.5793	22.105	0.9877	25.687	0.494	0.886

**Table 5:** Anti-inflammatory effect of F3, reference, and control in carrageenan-induced paw edema in rats.

Group	Treatment	Initial paw volume	Paw volume (mL)				Edema inhibition at 8 hs (%)
			1 hour	3 hours	5 hours	8 hours	
I	Control	1.15 ± 0.07	1.23 ± 0.02	1.59 ± 0.08	2.01 ± 0.03	2.28 ± 0.06	—
II	Reference	1.11 ± 0.08	1.19 ± 0.07	1.37 ± 0.05^∗^	1.50 ± 0.05^∗^	1.53 ± 0.01^∗^	75.83
III	F3	1.13 ± 0.05	1.18 ± 0.04	1.21 ± 0.02^∗^	1.32 ± 0.03^∗^	1.36 ± 0.04^∗^	92.64

Values are represented as mean ± SEM, *n* = 6 in each group, two-way ANOVA followed by Bonferroni's multiple comparisons, ^∗^ *p* < 0.05.

**Table 6:** The analgesic activity on rats measured by latency period (s) using the hot plate method.

	Latency (sec)			
Time (h)	0 h	0.5 h	1 h	3 h
Control	16.10 ± 3.36	16.75 ± 2.62	16.75 ± 3.2	16.10 ± 1.36
Reference	15.52 ± 1.00	23.12 ± 1.63	25.75 ± 1.7^∗^	21.75 ± 1.95
F3	15.75 ± 0.95	30.25 ± 3.59^∗∗^	36.50 ± 8.8^∗∗^	37.5 ± 2.40^∗∗^

Values are represented as mean ± SEM, *n* = 6 in each group, two-way ANOVA followed by Bonferroni's multiple comparisons, ^∗^ *p* < 0.05 and ^∗∗^ *p* < 0.001.

## Data Availability

The data used to support the findings of this study are included within the article.
